The article "Design and interactive performance of human resource management system based on artificial intelligence" was retracted in 2025. Reasons: compromised peer review; unreliable results or conclusions; concerns about the peer review; concerns about the article.

# Design and interactive performance of human resource management system based on artificial intelligence

**DOI:** 10.1371/journal.pone.0262398

**Published:** 2022-01-28

**Authors:** Yangda Gong, Min Zhao, Qin Wang, Zhihan Lv

**Affiliations:** 1 Business School, Hohai University, Nanjing, China; 2 Jiangsu Branch of China Mobile Group, Nanjing, China; 3 School of Data Science and Software Engineering, Qingdao University, Qingdao, China; Fuzhou University, CHINA

## Abstract

The purpose is to strengthen Human Resources Management (HRM) through information management using Artificial Intelligence (AI) technology. First, the selection criteria of the applicant’s resume during recruitment and the formulation standards of the contract salary are analyzed. Then, the resume information is extracted and converted into the data-type format. Besides, the salary forecast model in the HRM system (HRMS) is designed based on the Back Propagation Neural Network (BPNN), and network structure, parameter initialization, and activation function of the BPNN are selected and optimized. The experimental results demonstrate that the algorithm optimized by the Nadm has shown improved convergence speed and forecast effect, with 187 iterations. Moreover, compared with other regression algorithms, the designed algorithm achieves the best test scores. The above results can provide references for designing the AI-based HRMS.

## Introduction

With the socio-economic development, talents have become the mainstay of enterprise development, so more enterprises are competing for human resources rather than the traditionally narrower sense of labor resources. Furthermore, with structural informatization, enterprise data generation is increasing exponentially, which can no longer be efficiently handled using the manual Human Resource Management System (HRMS) [1]. Accordingly, the Information Management System (IMS) is employed to collect, store, manage, and analyze the exploding numbers of human resource data to improve the traditional enterprise Human Resource Management (HRM) [2]. In other words, HRM and Information Technology (IT) are combined in an attempt to establish an integrated HRMS to standardize the business process of Human Resource (HR) departments, centralize HR information, and enhance HRM transparency [3]. The quality of the HRMS will determine the enterprise performance and sustainable development. Therefore, it is urgent to establish a high-performance HRMS.

Numerous studies have shown that HRM efficiency can be uplifted by integrating IT. Therefore, this paper utilizes big data technology to manage and analyze HR data by designing a salary forecast model based on Artificial Intelligence (AI). The proposed model forecasts the salary by analyzing job applicants’ resumes from basic information, school, society, and enterprise factors. Then, the relevant parameters of the Back Propagation Neural Network (BPNN) are set and optimized to improve the forecast accuracy of the proposed model, and the model performance is tested through experiment. This paper innovatively integrates the BPNN into HRM to forecast employees’ salaries by analyzing their resumes to provide salary references for the HR department for the applicants and to promote enterprise development.

## Literature review

Abdullah et al. (2020) designed an enterprise cloud-based HRMS with 16 standard modules to solve HR problems using the CodeIgniter Web framework, which was then launched and deployed on the Amazon Web Service elastic computing cloud and used for an efficient enterprise HRM [4]. Necula and Strîmbei (2019) developed an architecture to semantically enrich data through data science and semantic web technology for talent training. The experimental results suggested that the classification effect of the proposed architecture was better than the commonly used regression analysis, Random Forest (RF), and Support Vector Machine (SVM), and the proposed architecture could effectively mark the resume data and use the semantic web to extract data information from the resume [5]. Jawad (2020) proposed a website-based HRMS to manage employee activity information, such as salary, registration, and promotion. The HRMS consisted of two parts: website design and database. Experimental results showed that the designed HRMS presented high performance and efficiency in employee information storage and management [6]. Qin et al. (2020) put forward a Recurrent Neural Network (RNN)-based applicant-job matching framework using job applicants’ perception ability, word-level semantic representation, and experience. This method could reduce the dependence on manual labor and improve employability. The information matching degree indicator was used to measure the importance of semantic representation and the contribution of job experience to job requirements [7]. Serje et al. (2018) used the occupational wage data from the International Labour Organization (ILO) to study econometric models of health workers’ income in different countries. They employed the selection model to analyze the skill and income data of health workers. The income of health workers varied in different countries and was negatively correlated with the country’s Gross National Product (GNP). The results could predict the cost of health care intervention and resource needs during sustainable development [8]. He et al. (2016) researched the cross-level relationship between salary differences and individual turnover intention. They investigated and analyzed employees’ annual objective salaries and self-reporting attitudes through the Questionnaire Survey (QS). Results demonstrated that the employee’s turnover intention and salary were positively correlated: the lower the salary was, the stronger the turnover intention was [9]. Shen et al. (2019) explored the organizational self-esteem, supervisory behaviors of communication between leaders, and restrictions on employee feedback behavior. They analyzed the employment behavior of different managers and employees through the hierarchical regression analysis and path analysis strategy. Results suggested that abuse supervision would directly affect employees’ turnover intention [10].

Briefly, the current research on HRMS mostly focuses on employee recruitment, registration, and management. Therefore, the salary forecast model is proposed for the BPNN-based HRMS to predict the salary of employees by analyzing the resume of candidates, thereby providing a check and balance mechanism for applicants and the enterprise interests.

## Method

### Salary forecast model in the BPNN-based HRM system

Usually, during the enterprise talent recruitment, qualified resumes are first picked out according to applicants’ age, educational background, work experience, and personal skills, which, traditionally, relies on manual selection. Thus, HR expertise knowledge, as well as some industrial common senses, are often required from the relevant personnel [11], where subjective human errors or prejudices might shut some outstanding talents out of the enterprise threshold. Then, the applicants are often informed of their possible salary range at the face-to-face interview stage, which might vary significantly per department and position [12]. Yet, the final salary is mostly determined by the department head after series of possible interviews and discussions, which, again, involves tremendous manual works that might, in turn, lead to deviations. There is an increasing voice calling for the elimination of such non-objective factors under the current competitive market environment.

Meanwhile, under the traditional HRMS, given limited HR personnel and countless applicants, resume selection is more a qualitative and speculative analysis process than an objective and scientific evaluation procedure. AI technology can well lend itself to such a predicament to help enterprises implement a salary forecast model, which can predict applicants’ salary based on their resumes from as early as the resume-selection stage and compares the forecast with their expected salary to provide further references [13]. The model-forecasted salary can be used as a benchmark salary for applicants, based upon which the actual salary can be reasonably adjusted considering the specific departmental and positional standards. An advantage of model-forecasted salaries is objectivity due to massive amounts of data calculation; on the other hand, the salary forecast model substantially reduces the workload of HR personnel and improves overall work efficiency [14].

The first step for salary forecast is the preprocessing of applicants’ resumes, after which the extracted structured information is used to train the salary forecast model against various data formats. The resume data can be classified as essential information and supplementary information, as shown in Fig 1, in which the resume is illustrated through hierarchically structured content. Common methods to extract information reasonably include the rule-based extraction, the Cascaded Hybrid Model, and the Conditional Random Field (CRF) extraction method.

**Fig 1:** Information level of resumes.

Employee salary determination is an intricate business that involves employee job specialty, as well as some subjective and objective factors, such as the nature of the enterprise. So is the salary forecast process that depends on the completeness of the resume information and the model performance to extract data features accurately and efficiently. The resume features division based on its content and formats read:

1. Personal factors: name, age, gender, phone number, and other information, divided according to the degree of association with salary forecast. For example, residence and birthplace will affect employment tenure; name, phone number, and email address are unique identifiers of the applicants; there may be special requirements on age and gender for specific positions [15].
2. School-related factors including school-time, alma mater, educational background, specialty, and awards. The alma mater and specialty can reflect an applicant’s learning ability and expertise skills, which also affect the salary forecast; awards are the manifestation of the applicant’s school performance and learning attitudes.
3. Social factors including served companies, positions, work hours, and length of service. Served companies and positions can reflect the level of personal abilities and skills. Length of service can reflect the mastery of relevant skills and personal adaptability. The number of served companies also affects the result of the salary forecast [16].
4. Enterprise factors are more closely related to the target enterprises. They are not included in the resumes, including the applying positions and occupation levels. Different enterprises in the same industry have different salary plans. The position applied to is the core of the salary forecast, which has a significant impact on the salary level. The occupational level is the requirement of salary level and the key to salary forecast [17].

Therefore, the salary demands of applicants should be forecasted from multiple aspects. Afterward, the character data extracted from the resume are converted into numerical data for subsequent data preprocessing and model training.

The salary forecast is a regression analysis process. The Neural Network (NN) in Machine Learning (ML) can be used as a salary regression forecast model, which is a parallel interconnected network composed of adaptive neural units and simulates the interaction process between the biological nervous system with the outside world. BPNN is the most common NN model. Theoretically, a 3-layer BPNN can approach a continuous function of arbitrary precision with a definite learning ability [18]. Yet, the network structure, parameter settings, and optimization algorithms will affect the NN training results and the salary model’s forecast effect. The learning process of the NN is the adjustment process of neuron parameters. BPNN’s error backpropagation process can adjust parameters. BPNN adopts a Gradient Descent (GD) strategy, which uses the target’s negative gradient direction as the search direction. During continuous iterations, the network parameters are updated, the model converges, and finally, the network parameters are adjusted [19].

BPNN contains a multi-layer signal feedforward NN, and the learning process is divided into two processes: forward propagation and directional propagation. The sample data enters the network from the input layer during the forward propagation, processed by the hidden layer and output from the output layer [20]. The error backward propagation process starts from the output layer, returns the results by layers in the reverse direction and the connection of neurons, and adjusts the neuron parameters in the path [21]. The processes of BPNN’s forward and backward propagation are illustrated in Fig 2.

**Fig 2:** The forward propagation and backward propagation processes in BPNN.

In the signal forward propagation process of the 3-layer BPNN, *x*_*i*_ represents the output of the input layer neuron, *l*_*j*_ denotes the output of the hidden layer neuron, and *z*_*k*_ indicates the output of the output layer neuron; *α*_*j*_ refers to the threshold of the hidden layer, and *β*_*k*_ stands for the threshold of the output layer; *w*_*ij*_ indicates the weight of the input layer to the hidden layer, and *v*_*jk*_ denotes the weight of the hidden layer to the output layer. The sample data are not processed in the input layer, and the output *l*_*j*_ of the *j*-th node in the hidden layer can be expressed as Eq (1).


$$l_{j}=f(net_{j})=f(\sum_{i}\left(w_{ij}x_{i}-\alpha_{j}\right))$$ (1)

The output *z*_*k*_ of the *k*-th node in the output layer reads:

$$z_{k}=f(net_{k})=f(\sum_{j}\left(v_{jk}l_{j}-\beta_{k}\right))$$ (2)

The output *z*_*k*_ of the output layer is the calculation of forward propagation. However, a gap exists between the generated forecast value and the actual value. The loss function *E* can serve as a standard to measure the error. The expression of loss function *E* reads:

E=C(θ;z) (3)

In Eq (3), *θ* = *θ*(*α*, *β*, *w*, *v*) represents all the network parameters, and *z* = (*z*_1_,*z*_2_,…*z*_*k*_) denotes the output vector [22]. BPNN uses a GD method to minimize the loss function in the continuous iteration process [23]. The calculation process is described as follows.

First, the connection weight gradient $\frac{\partial E}{\partial v_{jk}}$ of the output layer is calculated according to:

$$\frac{\partial E}{\partial v_{jk}}=\frac{\partial E}{\partial net_{k}}\cdot \frac{\partial net_{k}}{\partial v_{jk}}=\frac{\partial E}{\partial z_{k}}\cdot \frac{\partial z_{k}}{\partial net_{k}}\cdot \frac{\partial net_{k}}{\partial v_{jk}}$$ (4)

$$\frac{\partial E}{\partial v_{jk}}=C^{\prime }(\theta ;z){|}_{z_{k}}\cdot f^{\prime }(net_{k})\cdot l_{j}$$ (5)

The output error *δ*_*k*_, weight gradient $\frac{\partial E}{\partial v_{jk}}$, and threshold gradient $\frac{\partial E}{\partial \beta_{k}}$ of the output node are calculated as in Eqs (6)–(8), respectively:

$$\delta_{k}=-C^{\prime }(\theta ;z){|}_{z_{k}}\cdot f^{\prime }(net_{k})$$ (6)

$$\frac{\partial E}{\partial v_{jk}}=-\delta_{k}\cdot l_{j}$$ (7)

$$\frac{\partial E}{\partial \beta_{k}}=\delta_{k}$$ (8)

The connection weight gradient of the hidden layer $\frac{\partial E}{\partial w_{ij}}$ can be presented as:

$$\frac{\partial E}{\partial w_{ij}}=\frac{\partial E}{\partial net_{j}}\cdot \frac{\partial net_{j}}{\partial w_{ij}}=\frac{\partial E}{\partial l_{j}}\cdot \frac{\partial l_{j}}{\partial net_{j}}\cdot \frac{\partial net_{j}}{\partial w_{ij}}$$ (9)

$$\frac{\partial E}{\partial w_{ij}}=\sum_{k}C^{\prime }(\theta ;z){|}_{z_{k}}\cdot f^{\prime }(net_{k})\cdot v_{jk}\cdot f^{\prime }(net_{j})\cdot x_{i}$$ (10)

$$\frac{\partial E}{\partial w_{ij}}=\sum_{k}\delta_{k}\cdot v_{jk}\cdot f^{\prime }(net_{j})\cdot x_{i}=-f^{\prime }(net_{j})\cdot x_{i}\sum_{k}\delta_{k}\cdot v_{jk}$$ (11)

The calculations of the output error *γ*_*j*_, weight gradient $\frac{\partial E}{\partial w_{ij}}$, and threshold gradient $\frac{\partial E}{\partial \alpha_{j}}$ of the hidden layer read:

$$\gamma_{j}=f^{\prime }(net_{j})\cdot \sum_{k}\delta_{k}\cdot v_{jk}$$ (12)

$$\frac{\partial E}{\partial w_{ij}}=-\gamma_{j}\cdot x_{i}$$ (13)

$$\frac{\partial E}{\partial \alpha_{j}}=\gamma_{j}$$ (14)

Meanwhile, the learning rate *η* of each network layer can be adjusted to optimize the update step size and convergence speed of the iterative algorithm [24]. In BPNN, parameters are adjusted according to the negative gradient direction of the target. Assuming that the learning rate of each network layer is the same, then:

$$\Delta w_{ij}=-\eta \cdot \frac{\partial E}{\partial w_{ij}}=\eta \cdot \gamma_{j}\cdot x_{i}$$ (15)

$$\Delta \alpha_{j}=-\eta \cdot \frac{\partial E}{\partial \theta_{j}}=-\eta \cdot \gamma_{j}$$ (16)

$$\Delta v_{jk}=-\eta \cdot \frac{\partial E}{\partial v_{jk}}=\eta \cdot \delta_{k}\cdot l_{j}$$ (17)

$$\Delta \beta_{k}=-\eta \cdot \frac{\partial E}{\partial \beta_{k}}=-\eta \cdot \beta_{k}$$ (18)

$$\gamma_{j}=f^{\prime }(net_{j})\cdot \sum_{k}\delta_{k}\cdot v_{jk}$$ (19)

$$\delta_{k}=-C^{\prime }(\theta ;z){|}_{z_{k}}\cdot f^{\prime }(net_{k})$$ (20)

In Eqs (19) and (20), *f*() represents the activation function, and *c*() refers to the error function. Therefore, the gradient of the hidden layer parameters and the output layer parameters can be calculated by layers. This process is called backpropagation [25].

### Determining parameters of the salary forecast model

1. Network structure. Before BPNN can approach non-linear functions with arbitrary precision through its non-linear mapping, generalization, and fault tolerance capabilities, the network structure, activation function, and parameter initialization must be solved [26]. Since the salary forecast model processes multiple inputs while producing only one output, the number of input neurons must be determined. Based on the experimental analysis, the number of input and output neurons is set to 14 and 1, respectively. Since the hidden layer does not have a definite calculation equation, the hidden layer number is estimated first then determined through trial and error. The number of hidden layer neurons *n*_*h*_ can be determined according to:
$$n_{h}=\sqrt{n_{i}\cdot n_{o}}$$ (21)
$$n_{h}=\sqrt{n_{i}+n_{o}}+k,k\in [1,10]$$ (22)
  In Eqs (21) and (22), *n*_*i*_ represents the number of nodes in the input layer, and *n*_*o*_ denotes the number of nodes in the output layer [27].
2. Activation function. The activation function contains linear or non-linear functions used to solve linear problems and uncertain problems, respectively. The commonly used activation function Sigmoid function is expressed as Eq (23).
$$f(x)=\frac{1}{1+e^{-x}}$$ (23)
  The output result of this function is between (0, 1), and the function has differentiability and saturated nonlinearity, which can enhance the non-linear mapping ability of the network [28].
3. Parameter initialization. Parameter initialization will affect the training results and the convergence degree of the model. If the parameter setting is unreasonable, the model will fall near the local minimum during training and fails to converge. In the initial situation, the initial connection weight is accumulated, and the state of each neuron is 0. Neurons in the same layer should not be assigned the same weight; otherwise, the calculation result will be the same output [29]. Therefore, it is necessary to ensure that the connection weight is a random decimal number, and the value difference between each other is small. Hence, a good convergence speed will be obtained. This paper selects a Gaussian random number with a mean value of 0, and a standard deviation of $\sqrt{n_{in}}$ (*n*_*in*_ represents the number of neuron input connection weights), as well as a Gaussian random number with a mean value of 0, and a standard deviation of 1 as the weight and threshold parameters, respectively [30]. During algorithm training, the weight of the corresponding NN is reduced to minimize the recruitment discrimination caused by gender, age, and other factors.
4. Loss function. It can measure the error between the NN forecasted value and the actual value, which is the important criterion for training the learning model. Here, the objective function is calculated by quadratic Mean Square Error (MSE), as shown in Eq (24).
$$E\text{=}\frac{1}{2}{\left(y-z\right)}^{2}=C(\theta ;z)$$ (24)
  In Eq (24), *y* represents the objective function, and *z* denotes the output vector [31].
5. Optimization methods. BPNN has a simple structure and strong learning ability, but its complexity and performance are affected by the parameter initialization and network structure. Besides, given a flat error surface, oscillation will occur and affect the convergence speed. During the GD, the model easily falls into a local minimum and affects its forecast result. In the actual application, the convergence speed of BPNN needs to be optimized to avoid falling into a local minimum [32]. Common optimization methods include:
  1. In BPNN, the GD algorithm is applied to update the parameters in the backward propagation. According to the data bulk, the GD algorithm can be divided into Batch Gradient Descent (BGD) [33], Stochastic Gradient Descent (SGD) [34], and Mini-batch Gradient Descent (MBGD) [35].
  2. The last parameter change and the current parameter increment are connected by adding the former to the latter. This method of adding momentum to the parameter increment is called the additional momentum method, including the Momentum method and Nesterov Accelerated Gradient (NAG) method [36].
  3. The adaptive learning rate method dynamically adjusts the learning rate during the model training process to speed up convergence and reduce oscillations. Common adaptive learning rate optimization methods are Adagrad and RMSprop [37].
  4. Combining the additional momentum method and the adaptive learning rate method can obtain a hybrid optimization method that can optimize the GD. Such hybrid method has a fast convergence speed and fewer oscillations, including Adaptive Moment Estimation (Adam) and Nesterov-accelerated Adaptive Moment Estimation (Nadam) [38].

In summary, the ratio of the number of neurons in the input layer, the hidden layer, and the output layer is 14:15:1 in the designed 3-layer BPNN. The activation function is a Sigmoid function, while the error function is a quadratic MSE function. MBGD and Nadam optimization algorithms are used to optimize the model, and the BPNN parameters and experimental environment are displayed in Tables 1 and 2. Therefore, the output errors *δ*_*k*_ and *γ*_*j*_ of the output layer and the hidden layer are calculated according to:

**Table 1:** BPNN parameter setting.

Parameter	Value	Parameter	Value
Learning rate	0.1	Number of network layers	4
Maximum number of training	10	Number of input layer neurons	14
Accuracy required by the training	0	Number of hidden layer neurons	15
Minimum gradient requirement	1.00E-10	Number of output layer neurons	1
Training iteration process displayed	25	GD algorithm	MBGD algorithm
Maximum training time	inf		Nadam algorithm
Momentum factor	0.9	Loss function	Quadratic mean square function
		Activation function	Sigmoid function

**Table 2:** Experimental hardware and software environment.

Hardware environment	CPU	Intel Xeon E5-2640 v4 @2.40GHz	Software environment	Operating system	Ubuntu 14.04
	Graphics Processing Unit (GPU)	NVIDIA TITANX (pascal)		Software	Python 2.7
	RAM +Internal memory	16GB+256GB			


$$\delta_{k}=-(y_{k}-z_{k})\cdot z_{k}\cdot (1-z_{k})$$ (25)

$$\gamma_{j}=l_{j}\cdot (1-l_{j})\cdot \sum_{k}\delta_{k}\cdot v_{jk}$$ (26)

In Eqs (25) and (26), *y*_*k*_ and *z*_*k*_ represent the target value and output value of the *k*-th node. The salary forecast model’s training process based on BPNN is shown in Fig 3 [39].

**Fig 3:** The training process for the salary forecast model.

### Introduction to experimental samples

Because salary forecast belongs to a multiple-input-single-output mapping process, effective salary forecast results can be obtained by considering different influencing factors of salary like the model’s output and optimizing the influence weight of each factor in the model through training. The information in the resume library of an enterprise is analyzed to verify the effect of the designed model. The number of samples is 1,000, of which the number of recruits is 298, the number of rejections is 702, and each resume has a corresponding salary status. Data characteristics of the resume include age, salary, gender, the highest academic credential, major, marital status, job position, position applied, work experience, and length of service. Since the salary forecast model structure is affected by the training samples and model parameters, the most suitable parameter settings are obtained by continuously adjusting the model parameters. Recruitment bias caused by factors such as gender and age may arise during employee recruitment. However, in the present work, the resume data of the enterprise after successful recruitment is used so that the work does not directly consider the possible moral hazard. Among the risks, the generated salary forecast model also meets the enterprise’s recruitment requirements. Therefore, the research results do not consider the possible moral hazard. To better compare the classification effect of the classifier, the following indicators are employed to evaluate the classification effect of the classifier. Among them, *TP* refers to the proportion of resumes correctly classified as entry, *FP* denotes the proportion of resumes incorrectly classified as entry, *TN* indicates the proportion of resumes correctly classified as non-entry, and *FN* represents the proportion of resumes incorrectly classified as the entry.

1. Precision refers to the total proportion of positive samples correctly classified by the classifier.
$$Precision=\frac{TP}{TP+FP}$$ (27)
2. *Recall* in Eq (28) indicates the proportion of positive samples that are correctly predicted.

$$Recall=\frac{TP}{TP+FN}$$ (28)

## Results and discussion

### Parameter selection

According to the empirical equation, the number of neurons is in the range of [5, 14]. Hence, the model with several neurons between [3, 16] is trained and tested. The number of samples used is 1,000, with 500 in the training set and 500 in the validation set. The hidden layer neurons are trained 30 times to obtain the average result. The number of iterations is set at 1,000, with the training loss accuracy E<0.01. The training results are displayed in Fig 4.

**Fig 4:** Comparison of training results of different numbers of neurons in the hidden layer.

According to Fig 4, when the number of neurons in the hidden layer is 14, the model’s training loss is the smallest, which is 0.009914. When the number of neurons is 15, the number of iterations and the model’s verification loss are the smallest, of 64 and 0.010511, respectively. Therefore, the number of nodes in the input layer, the hidden layer, and the output layer of the designed BPNN is 14, 15, and 1, respectively. Such a structure can accelerate the model’s running speed and reduce the verification loss and training loss.

The effect of the optimization algorithm on the model is verified through the Leave-One-Out (LOO) method. The sample-set with 1,000 samples is divided into a training set with 900 samples and a test set with 100 samples. The number of cycles is set to 10,000, or the training is stopped when the training loss accuracy E is less than 0.005. The convergence speed of the model optimized by different algorithms is shown in Fig 5; the comparison of training results is displayed in Fig 6.

**Fig 5:** Comparison of the convergence speed of different optimization methods.

**Fig 6:** Comparison of training results of different optimization methods.

As shown in Fig 5, among various optimization algorithms, Adam and Nadm have faster convergence speeds than other optimization algorithms, which can quickly converge to the minimum and reduce the model’s running time. Furthermore, the convergence effect of Nadm is better than that of Adam. According to the training results comparison of six algorithms, the test scores and training losses of various optimization algorithms are close. However, there are noticeable differences in the number of training cycles. SGD has the largest number of training cycles, of 3,228 times. In contrast, Nadm has the minimal training cycles of 187 times. Therefore, among the various NN GD algorithms, the hybrid optimization algorithm Nadm presents the best optimization effect and convergence speed. Hence, Nadm is chosen as the GD optimization algorithm for the salary forecast model.

### Analysis of salary relevance

It has been argued that salary level might somehow reflect the relevance between talent supply and recruitment positions. This section selects 10,000 pieces of enterprise recruitment data, including the lowest salary, highest salary, and average salary, location, company size, financing, education level, work experience, and job type. First, the relevance among different influencing factors is analyzed using the Pearson correlation coefficient method, and the results are shown in Fig 7. Fig 7 reveals that the relevance between salary is the strongest, and the relevance among education level, job type, and work experience and salary is also stronger than other influencing factors. Therefore, salary is taken as the dependent variable with the influencing factors including job type, work experience, and education level as the independent variable, and the analysis results are shown in Fig 8.

**Fig 7:** Analysis of salary relevance.

**Fig 8:** The relationship between dependent variables and salary. a) Job type; b) Work experience; c) Education level.

Fig 8A suggests that there is a certain relationship between job type and salary. The salary of different jobs varies much. The salary range of data risk jobs and products is 15-25k/month. The development of the Internet in recent years has made the income of related industries continue to rise. Operation positions and design positions are affected by personnel, and the salary will also change. Fig 8B indicates that the salary will continue to improve with the accumulation of work experience. The salary will not change much within three years, but will increase after three to five years, and will increase significantly after five to ten years. The maximum monthly salary can reach more than 40 k/month. Hence, after several years of work experience, employees can get a higher salary. Fig 8C shows that with the improvement of education level, the salary also rises. The salary of undergraduates is 50% higher than that of college students. The salary of masters and doctors is much higher than that of other education levels, and the salary ceiling of doctors is higher. To sum up, job type, work experience, and education level are the main factors that affect salary, and the different influencing factors will also affect salary. But in general, the higher the education level is, the richer the work experience is, and the more likely the employees in popular positions are to get a high salary.

### Performance test

The resume information status of the experimental sample is summarized in Fig 9. The salary forecast model based on BPNN is applied to fit the salary data to verify its actual forecast effect, and the results are shown in Fig 10. Common regression algorithms are adopted for comparative simulations, including Linear, Polynomial, Ridge, Lasso, and ElasticNet. The ratio of the correct number of samples output by different models to all samples is taken as the model’s score. The scores of the training process and testing process are presented in Fig 11. The number of samples in the training set used for model training is 900, and the number of samples in the test set is 100. Six experiments are carried out on each model and the average value is taken as the final result.

**Fig 9:** Resume information distribution. a) Applicant department status; b) Resume information status.

**Fig 10:** The fitting effect of Nadm-optimized salary forecast model.

**Fig 11:** Comparison of salary forecast results of different algorithms.

Fig 9 presents that the recruitment data involves different job types, and the data content includes salary level, gender, education level, and other information. According to Fig 10, the BPNN-based salary forecast model optimized by the Nadm gradient has an excellent fitting performance. However, some errors still exist. The reason may be that the data are normalized during the model training process, resulting in errors in the calculation results. However, the overall error is acceptable. As shown in Fig 11, the Nadm gradient optimization model has the highest test score than other algorithms.

### Performance comparison

BPNN is employed to analyze the establishment information to obtain the forecasted salary and compare the salary level of the sample database from precision and recall rate. The forecast results of the LSTM network, GRU network, Bi-LSTM network, and Bi-GRU network are compared, as illustrated in Fig 12.

**Fig 12:** Comparison of salary forecast results of different NN algorithms.

As shown in Fig 12, the precision and recall rate of BPNN optimized by the GD algorithm for salary forecast is above 0.9, which is better than the forecast results of the LSTM network, GRU network, Bi-LSTM network, and Bi-GRU network. Hence, the actual effect of the designed salary forecast model can provide better accuracy than similar models. Thus, during the actual application, a desirable salary can be provided to applicants by analyzing their resumes. The results can provide a theoretical reference for establishing a reasonable employee salary system.

In summary, the designed salary forecast algorithm based on the BPNN model uses a network structure with 14:15:1 (input layer: hidden layer: output layer) of the number of neurons. Besides, the Nadm gradient optimization algorithm is used to optimize the model to get a faster convergence speed and excellent forecast effect. Compared with other regression algorithms, the algorithm used here has the best forecast effect and test score. The actual forecast results also show that the salary forecast model can provide desirable salaries for applicants. Therefore, the designed salary forecast algorithm can apply to forecast the salary in the HRM system.

## Conclusion

This work aims to build an intelligent HRMS and improve the efficiency of HRM. A Human-Computer Interaction (HCI)-based HRMS is designed using AI technology to strengthen enterprises’ management and development capabilities. First, J2EE is employed to design a modularized HRMS. Second, the Artificial Neural Network (ANN) is adopted to optimize the HRMS, and the salary forecast module is implemented to effectively judge the applicants’ ability according to the resume and industry information, thereby offering a reasonable salary. Eventually, the performance of the designed salary prediction model of the HRMS is tested and analyzed. The experimental results demonstrate that the network structure, parameter settings, and gradient optimization algorithm will affect the model’s forecast structure. Tests prove that the Nadm gradient optimization algorithm can effectively improve the model’s convergence speed and actual fitting effect. Compared with other algorithms, the model optimized by Nadm has optimal test scores. Therefore, the proposed algorithm can be applied to the salary forecast of the HRM system. However, there are still some shortcomings. The salary of applicants might be affected by many factors in real life, but this paper conducts the correlation analysis only on several main influencing factors, so the proposed salary forecast model is relatively simple, with a weak data feature processing ability. In the research process, the model has been optimized to further reduce the impact of potential recruitment discrimination on the output of the model. In the follow-up research, it is worth considering more possible influencing factors to enhance the model forecast ability and accuracy.

## Supporting information

S1 Data (ZIP)
